# Correlation between Serum Levels of High Mobility Group Box-1 Protein and Pancreatitis: A Meta-Analysis

This article has been retracted.

**DOI:** 10.1155/2015/430185

**Published:** 2015-01-28

**Authors:** Yan Lin, Lian-Jie Lin, Yu Jin, Yong Cao, Ying Zhang, Chang-Qing Zheng, Jia-Li Liu, Sheng-Li Yang

**Affiliations:** ^1^Department of Gastroenterology, Shengjing Hospital, China Medical University, Sanhao Street No. 36, Heping District, Shenyang 110001, China; ^2^Department of Oncology, Renji Hospital, Shanghai Jiao Tong University, Shanghai 200000, China

## Abstract

*Background*. Aberrant expression of high mobility group box-1 protein (HMGB1) contributes to the progression of various inflammatory diseases. This meta-analysis focused on the clinical significance of serum HMGB1 levels in pancreatitis patients, with the goal of building a novel diagnostic score model. *Method*. We conducted a meta-analysis by searching in the PubMed, Embase, Web of Science, Cochrane Library, CISCOM, CINAHL, Google Scholar, China BioMedicine (CBM), and China National Knowledge Infrastructure (CNKI) databases without any language restrictions. Studies were pooled and standard mean difference (SMD) and its corresponding 95% confidence intervals (95% CIs) were calculated. Version 12.0 STATA software was used for statistical analysis. *Results*. We performed a final analysis of 841 subjects from 12 clinical case-control studies. The meta-analysis results showed a positive association between serum HMGB1 levels and the progression of pancreatitis. In the subgroup analysis by country, high serum level of HMGB1 may be related to pancreatitis progression in China, Korea, Hungary, and Japan populations (all *P* < 0.05). *Conclusion*. The present meta-analysis indicated that serum HMGB1 level was statistically elevated in patients with pancreatitis, and thus serum levels of HMGB1 could be determined to be a useful biomarker for pancreatitis patients.

## 1. Introduction

Pancreatitis is an inflammatory disorder that causes irreversible anatomical changes and damage, including infiltration of inflammatory cells, fibrosis, and calcification of the pancreas with destruction of the glandular structure, and thereby affects normal digestion and absorption of nutrients [1]. Abdominal pain is a major clinical challenge in pancreatitis, present in up to 90% of the patients, and is the primary cause of hospitalization [2]. There are two types of pancreatitis, namely, the chronic and acute types; chronic pancreatitis is a clinical challenge, with persistent or recurrent abdominal pain as the most compelling symptom that drives patients to seek medical care [3, 4]. Acute pancreatitis is a mild, self-limited disease and is a common cause of acute abdominal pain [5]. Severe acute pancreatitis is characteristic of a serious pathogenetic condition with high incidence of complications and 20%–30% of mortality, and there is still no breakthrough in treatment [6, 7]. An estimated 210,000 new cases of acute pancreatitis occur each year in the United States [8]. In Germany, the incidence of this disease is rising and has now reached 23 cases per 100,000 persons per year [9]. Some 20% to 30% of patients develop severe disease manifested by pancreatic necrosis, abscess or pseudocysts, and extrapancreatic complications such as vital organ dysfunction [5]. Furthermore, about 20% of cases of severe acute pancreatitis are necrotizing disease, which accounts for nearly all the morbidity and death associated with acute pancreatitis [10]. The etiology of pancreatitis is multifactorial and the risk factors include alcohol and nicotine consumption, hereditary factors, efferent duct obstructions, immunological factors, or rare metabolic disorders [11]. Conventional biomarkers of pancreatitis such as CA19-9 and carcinoembryonic antigen may also be elevated in benign conditions or in cancers; hence their inadequate sensitivity and specificity restricted the use of those markers in the early diagnosis of pancreatitis [12–14].

High mobility group box-1 protein (HMGB1), also named amphoterin, is a DNA-binding intranuclear protein with the function of proper transcriptional regulation and gene expression and takes part role in DNA replication and repair, neurite outgrowth, and cell motility [15, 16]. In clinical practice, it has been found that, as an extremely mobile protein, HMGB1 has a significant role in both nucleic acid-activated innate immune responses and macrophage-related inflammatory reaction [17, 18]. In particular, it has been studied that HMGB1 may bind to all immunogenic nucleic acids and mediate the immune system through stimulating the transcription of type 1 IFN, IL-6, and RANTES from immune cells [18]. In addition, inflammatory function of HMGB1 has been further discovered that HMGB1 may be capable of prolonging and sustaining inflammatory processes by inducing macrophages to release cytokines and inflammatory mediators such as TNF-*α*, IL-1*α*, IL-1*β*, and IL-8 when released into an extracellular environment [19]. In particular, numerous studies have emphasized the important role of proinflammatory cytokines in the mechanism that severe acute pancreatitis develops systemic inflammatory response syndrome, multiple organ failure, and even death [7, 20]. For instance, increased HMGB1 levels were found in the plasma of patients with chronic lymphocytic leukemia when compared to healthy controls, and the concentration of HMGB1 is suggested to be correlated with the absolute count of lymphocyte [21]. In recent studies, an increased serum level of HMGB1 has been shown in progression of many acute and chronic inflammatory diseases, such as sepsis, acute lung injury, rheumatoid arthritis, and disseminated intravascular coagulation, suggesting that HMGB1 may have a large influence on the development and evolution of malignant processes by promoting cell migration, modulating the adhesive properties, and stimulating tumor neoangiogenesis [7, 12, 22]. Currently, with the increasing studies on pancreatitis, several findings have revealed that HMGB1 may be secreted by necrotic cells of the injured pancreas and other damaged organs, which may accelerate the inflammation and may be attributed to tissue injury and organ failure in acute pancreatitis [23–26]. Moreover, it has demonstrated that the serum level of HMGB1 may be higher in late-stage pancreatic ductal adenocarcinoma (PDAC) than that in early-stage PDAC [12, 25]. Taking the above findings into consideration, we hypothesized that serum HMGB1 level may be associated with the diagnosis and prognosis of pancreatitis [24–27]. However, some studies insisted that serum levels of HMGB1 possibly have no correlation with the severity or outcome of acute pancreatitis as the difference of serum HMGB1 level appears not significant in patients with or without organ dysfunction [28, 29]. Consequently, this meta-analysis was performed to evaluate the diagnostic and prognostic value of serum HMGB1 level in patients with pancreatitis.

## 2. Materials and Methods

### 2.1. Search Strategy

Correlated studies were identified by searching PubMed, Embase, Web of Science, Cochrane Library, CISCOM, CINAHL, Google Scholar, China BioMedicine (CBM), and China National Knowledge Infrastructure (CNKI) databases comprehensively for all published articles which assessed the relationships between serum levels of HMGB1 and pancreatitis from July 24, 2006, to April 30, 2014, using the following search terms (“Pancreatitis” or “chronic pancreatitis” or “acute pancreatitis”) and (“HMGB1 Protein” or “HMGB1” or “HMG 1 Protein” or “HMG1” or “Amphoterin” or “Heparin-Binding Protein p30” or “high-mobility group box 1” or “High mobility group box protein 1”). No limitation was placed on the language of the article in English and Chinese. Additional potential relevant articles were further retrieved through a manual search of references from original reports.

### 2.2. Selection Criteria

Any randomized intervention case-control studies that involved the association of serum levels of HMGB1 with pancreatitis as a primary outcome were initially taken into consideration. At the time of their admission, studies that had patients diagnosed with different grades of pancreatitis were confirmed by the Japanese severity score (JSS), a criterion for clinical diagnosis and grading severity formulated by the Intractable Diseases of Pancreas, Japan Ministry of Health, Labor and Welfare. Studies that did not provide the number of pancreatitis cases, or sufficient information about serum HMGB1 expression levels, were excluded. Articles with more than 30 recorded cases of pancreatitis were included in the initial review. Studies that did not indicate the number of cases nor provided sufficient information about HMGB1 expression levels were excluded. If more than one study by the same author using the same case series was published, both the study with the largest sample size and the most recent publication were included.

### 2.3. Data Extraction

From each eligible article, two investigators abstracted information independently using a standardized protocol and data recording form and reached a consensus on all the items through discussion of disagreements. Information, such as surname of first author, year of publication, source of publication, study type, study design, sample size, age, sex, ethnicity and country of origin, detection method of HMGB1 serum levels, and expression levels, was collected from each study. Due to subjects from different ethnicities, information was extracted separately and stratified into two groups, the Asians and Caucasians. All authors approved the final list of these enrolled studies.

### 2.4. Quality Assessment

To decide whether the study in question is of high quality, the two reviewers used a set of predefined criteria, the Newcastle-Ottawa Scale (NOS) criteria, to assess the studies independently [37]. The NOS criteria are scored based on three aspects: (1) subject selection: 0~4; (2) comparability of subject: 0~2; (3) clinical outcome: 0~3. Total NOS scores range from 0 (lowest) to 9 (highest). According to the NOS scores, the included studies were classified into two levels: low quality (0–6) and high quality (7–9), respectively. Any discrepancies between the two reviewers on NOS scores of the included studies were resolved by discussion and consultation with a third reviewer.

### 2.5. Statistical Analysis

In order to supply quantitative evidence of all selected studies and minimize the variance of the summary, we conducted the current statistical meta-analyses utilizing a random-effects model (DerSimonian and Laird method) or a fixed-effects model (Mantel-Haenszel method) with inverse-variance (SE) weighting of individual study results under the situation where data from independent studies could be combined. Random-effects model was used when heterogeneity exists among studies, while fixed-effects model was used when there was no statistical heterogeneity. The summary standardized mean difference (SMD) with 95% confidence intervals (CIs) was calculated for case versus control category of HMGB1 serum levels by the use of *Z* test. The subgroup meta-analyses were also conducted by country and the degree of disease to explore potential effect modification, and heterogeneity across the enrolled studies was evaluated by Cochran's *Q*-statistic (*P* < 0.05 was regarded as statistically significant) [38]. As a result of low statistical power of Cochran's *Q*-statistic, *I* ^2^ test was also measured to reflect the possibility of heterogeneity between studies [39]. To evaluate the influence of the individual data set on the pooled SMD, a one-way sensitivity analysis was conducted by deleting one study at a time. The funnel plot was constructed to assess if publication bias affects the validity of the estimates. The symmetry of the funnel plot was further evaluated by Egger's linear regression test [40]. All tests were two-sided and a *P* value of <0.05 was considered statistically significant. To make sure that the results are credible and accurate, two investigators entered all information in the STATA software, version 12.0 (StataCorp, College Station, TX, USA), separately and arrived at an agreement.

## 3. Results

### 3.1. Baseline Characteristics of Included Studies

The original search yielded a total of 131 papers related to the searched keywords. The flow chart of the study selection process is summarized in Figure 1. Through the step of screening the title, key words, and abstracts 53 of these articles were excluded (3 were duplicates, 10 were letters, reviews, or meta-analysis, 16 were not human studies, and 24 were not related to research topics). Full-text articles from 78 articles were reviewed and an additional 63 trials were excluded (12 were not case-control study, 18 were not relevant to HMGB1 serum level, and 33 were not relevant to pancreatitis), leaving 15 studies for further review. Of these, 3 were excluded for not providing sufficient data; therefore, 12 papers [12, 24, 27–36], which included a total of 841 subjects (455 patients with pancreatitis and 386 healthy controls), were finally found to conform to our inclusion criteria. From 2001 to 2014, the number of articles selected from those electronic databases was shown in Figure 2. Publication year ranged from 2006 to 2013, and no related studies on HMGB1 in pancreatitis were found prior to 2006. All articles were case-control studies that assessed the relationship of HMGB1 serum levels and pancreatitis in Asian populations (11 studies) and Caucasian populations (1 study). Detection method used in all the papers included in this meta-analysis is enzyme linked immunosorbent assay (ELISA). All quality scores of the enrolled papers were higher than 7 (high quality).  Table 1 summarized the characteristics and methodological quality of the enrolled studies.

### 3.2. Serum Levels of HMGB1 in Pancreatitis

A total of 12 case-control studies referred to the HMGB1 serum levels in pancreatitis. Our meta-analysis results identified a positive association between HMGB1 serum levels and the progression of pancreatitis (SMD = 3.42, 95% CI: 2.82–4.03, *P* < 0.001). The random-effects model was used because of existing heterogeneity (*P* < 0.001). The major results of the correlations between the levels of HMGB1 and pancreatitis are supplied in Figure 3. Subgroup analysis based on country implied that high level of serum HMGB1 may be the main risk factor of pancreatitis progression in China, Korea, Hungary, and Japan populations (all *P* < 0.05) (Figure 4). Further subgroup analyses by the degree of disease showed positive association between the levels of HMGB1 and pancreatitis progression in all the subgroups (all *P* < 0.05).

### 3.3. Sensitivity Analysis and Publication Bias

A sensitivity analysis's results showed that the overall statistical significance does not change when any single study was omitted. Therefore, the current meta-analysis data is relatively reliable and credible (Figure 5). The graphical funnel plots of those 12 studies are slightly asymmetrical, and Egger's test showed that there is publication bias on the positive association of HMGB1 serum levels with the progression of pancreatitis in this meta-analysis (*t* = 7.53, *P* < 0.001) (Figure 6).

## 4. Discussion

We performed this meta-analysis to observe the alterations of HMGB1 plasma concentrations in patients with pancreatitis and to explore its relationship with the severity of pancreatitis, revealing its diagnostic and prognostic ability for pancreatitis. The findings in our study have indicated that serum HMGB1 levels were significantly increased in patients with pancreatitis and were correlated with disease severity, suggesting that serum HMGB1 concentrations can be regarded as an important cytokine mediator in the pathogenesis of severe acute pancreatitis. Nevertheless, the exact mechanism by which serum level of HMGB1 is related to the development and progression of pancreatitis is not fully understood at present. It was well established that various proinflammatory cytokines may play very crucial roles in the development of pancreatitis, which may accelerate the deterioration of pancreatitis into systemic inflammatory response syndrome and may result in organ failure or even death [41]. As a late-acting proinflammatory cytokine, HMGB1 mediates many crucial pathological processes such as inflammation, cell migration, and tissue regeneration [42]. Furthermore, HMGB1 may be involved in the development and evolution of malignant processes through its ability to promote cell proliferation and migration, modulate the adhesive properties, and stimulate tumor neoangiogenesis [43]. In addition, abnormal-activated pancreatin damages adjacent pancreatic cells and leads to local infiltration of inflammatory cells, and activated inflammatory cells such as macrophage, neutrophil, and pancreatic acinar cells can produce and release inflammatory cytokines including HMGB1 [12]. Notably, HMGB1 is actively secreted from monocytes or macrophages in response to proinflammatory stimuli, such as IL-1 and TNF-*α*, and it can also be passively released by necrotic cells that will induce inflammation; thus HMGB1 may be involved in the pathophysiological process of various infectious diseases including pancreatitis and enhance the inflammatory response [23, 44]. Furthermore, extracellular HMGB1 can induce the release of proinflammatory mediators, which can result in highly increased serum levels of proinflammatory cytokines, and then cause the activation of immune system, as well as invasion by inflammatory cells, thereby prolonging and sustaining inflammatory processes [42]. In this regard, the rising degree of HMGB1 serum level can amplify the inflammation and may contribute to tissue injury and organ failure and may be closely associated with the severity of pancreatitis and its development. Zhang et al. have demonstrated that HMGB1 was upregulated in patients with severe acute pancreatitis, which may seem to act as a late cytokine mediator in the pathogenesis of severe acute pancreatitis [7]. Yang et al. have indicated that the HMGB1 serum level was obviously increased in severe acute pancreatitis patients and the death patients during the hospitalization showed a significantly high serum HMGB1 level, implying that the elevated serum HMGB1 level may be a potential predictor in the development of pancreatitis [29]. Meanwhile, Wang et al. have observed that the serum level of HMGB1 was significantly increased in the second day of hospitalization when compared with that in the first day of hospitalization, and the elevated serum level of HMGB1 in the patients with acute pancreatitis maintained a high level along with the length of stay, indicating that the upregulated HMGB1 level may be connected with the development of pancreatitis [32].

To investigate the exact relationships between the HMGB1 serum level and the development and progression of pancreatitis, we also carefully carried out stratified analysis on the basis of country and the severity of pancreatitis. Our findings of country-stratified analysis have revealed that the plasma concentrations of HMGB1 were significantly increased in patients with pancreatitis in China, Korea, Hungary, and Japan populations, implying that country differences may not be the potential heterogeneity source. Further subgroup analysis based on the severity of pancreatitis has indicated that there were positive associations between the serum levels of HMGB1 and all the progression of pancreatitis including SAP, mild acute pancreatitis (MAP), acute pancreatitis (AP), and chronic pancreatitis (CP), suggesting that serum HMGB1 levels may serve as a major risk factor of pancreatitis progression. In brief, our results indicate that an elevated HMGB1 serum level was closely correlated with the occurrence and progression of pancreatitis; thus it can act as a potential diagnostic and prognostic predictor for pancreatitis.

Meanwhile, there did exist some limitation in the current meta-analysis which should be noted. Firstly, there is the possible existence of biases. Although we performed a methodological assessment of those studies to avoid some selection biases, there was a highly significant heterogeneity among the 12 evaluable articles which may be attributed to the fact that the technique of detecting HMGB1 may not be comparable among studies. Secondly, there is the potential publication bias in this study, since we did not take several unpublished articles and abstracts into account due to their unavailability. In addition, we only picked up eligible English or Chinese studies language in this meta-analysis, while other languages were excluded based on language criteria, which may also introduce bias and affect the findings in our study. A third potential limitation is that our meta-analysis may still be underpowered to acquire original data from the included studies. Finally, serum levels of HMGB1 may also elevate in other cancers that may have false positive impression of our results and hence influence the credibility and reliability of our findings. Despite the above limitations, this is the first example of meta-analysis on the association of serum HMGB1 levels with the development of pancreatitis. With the application of a statistical approach to combine the results from multiple studies in our meta-analysis and to achieve strong objectivity, all the research methods were carried out on strict inclusion and exclusion criteria, suggesting that obtained information may approximate the actual results.

In brief, this meta-analysis indicated an elevation of HMGB1 serum level in pancreatitis patients, demonstrating that the increased serum level of HMGB1 may contribute to an aggressive progression of pancreatitis. The early detection of serum levels of HMGB1 and approaches involving the inhibition of HMGB1 may help clinicians to determine valuable therapeutic strategies for pancreatitis patients.

## Figures and Tables

**Figure 1:** Flow chart shows study selection procedure. Twelve clinical case-control studies were included in this meta-analysis.

**Figure 2:** The distribution of topic-related literature in the electronic database over the last decade. The bar graph means the distribution of all related topics, and the line graph represents all the papers used in the review.

**Figure 3:** Forest plot for the difference of serum HMGB1 levels between pancreatitis patients and control subjects. The dots in these figures represent the results in each included study, and the diamonds in these figures represent the results of our study.

**Figure 4:** Subgroup analyses for the difference of serum HMGB1 levels between pancreatitis patients and control subjects. The dots in these figures represent the results in each included study, and the diamonds in these figures represent the results of our study.

**Figure 5:** Sensitivity analysis of the summary odds ratio coefficients for the difference of serum HMGB1 levels between pancreatitis patients and control subjects. The circle represents the summary odds ratio of remaining articles calculated by deleting the corresponding article, and the line segment represents the 95% confidence intervals.

**Figure 6:** Funnel plots for the difference of serum HMGB1 levels between pancreatitis patients and control subjects.

**Table 1:** Main characteristics and methodological quality of all eligible studies.

First author	Year	Country	Ethnicity	Sample size		Gender (M/F)		Age (years)		Method	Disease	NOS score
				Case	Control	Case	Control	Case	Control			
Yang [29]	2013	China	Asians	72	72	40/32	38/34	40.2 ± 11.8	40.6 ± 10.8	ELISA	SAP	8
Shi [30]	2013	China	Asians	79	50	—	29/21	—	44.0 ± 5.0	ELISA	SAP/MAP	6
Qu [28]	2013	China	Asians	32	40	20/12	25/15	41.9 ± 12.3	40.9 ± 11.9	ELISA	SAP/MAP/AP	7
Zhang [31]	2012	China	Asians	38	30	18/20	16/14	23~89	21~69	ELISA	SAP/MAP	7
Wang [32]	2012	China	Asians	24	20	16/8	13/7	44.8 ± 13.3	42.3 ± 10.5	ELISA	SAP/MAP	7
Chung [12]	2012	Korea	Asians	25	25	15/10	15/10	55.7 ± 9.5	54.2 ± 10.4	ELISA	CP	7
Yu [33]	2011	China	Asians	32	30	17/15	18/12	29~65	28~62	ELISA	SAP/MAP	7
Xia [34]	2011	China	Asians	33	51	16/17	26/25	36~90	21~76	ELISA	SAP/MAP	8
Lu [35]	2011	China	Asians	35	20	20/15	12/8	60.0 ± 16.5	42.0 ± 17.0	ELISA	SAP/MAP/AP	7
Lu [36]	2010	China	Asians	10	20	6/4	10/10	41.7 ± 3.2	41.6 ± 1.9	ELISA	SAP/MAP	6
Kocsis [24]	2009	Hungary	Caucasians	30	20	19/11	—	—	—	ELISA	SAP/MAP	5
Yasuda [27]	2006	Japan	Asians	45	8	13728	—	50.0 ± 1.9	—	ELISA	SAP	6

M: male; F: female; ELISA: enzyme linked immunosorbent assay; NOS: Newcastle-Ottawa Scale; AP: acute pancreatitis; SAP: severe acute pancreatitis; MAP: mild acute pancreatitis; CP: chronic pancreatitis.
